This article has been retracted.

# Clinical Rehabilitation Nursing of Patients with Chronic Obstructive Pulmonary Disease Based on Intelligent Medicine

**DOI:** 10.1155/2022/8021967

**Published:** 2022-09-19

**Authors:** Lingyan Zhao, Liyan Chu

**Affiliations:** Qingdao University, Qingdao, 266021 Shandong, China

## Abstract

Chronic obstructive pulmonary disease (COPD) is a respiratory disease that can be treated and prevented. The purpose of this paper is to conduct a meta-analysis of clinical rehabilitation nursing of COPD patients based on intelligent medical care by constructing a suitable model so as to make the research on clinical nursing of COPD patients more effective. This paper first introduced the intelligent medical system, analyzed the clinical rehabilitation nursing of COPD patients, established the SCNet model suitable for this paper, and then used statistical algorithms to carry out the meta dynamic analysis of the clinical rehabilitation nursing for COPD patients. Through the analysis of the current situation of medical equipment and the comparison of models and statistical analysis, the experimental results showed that the pulmonary function indexes of the pulmonary rehabilitation treatment group and the conventional treatment group were improved after treatment compared with before treatment. Although on specificity metrics SCNet did not perform the best, it was about 1% lower than the best baseline model. However, the comprehensive performance of the SCNet model on Acc, Sen, F1-Score, and AP indicators showed that the model SCNet proposed in this paper had certain advantages, which was helpful for the clinical rehabilitation care of patients with COPD and could better assist doctors in treatment.

## 1. Introduction

With the development of medical technology, the term intelligent medical care appears in front of the public. In the meantime, China's medical care has developed. Most medical bachelors will also invest a lot of energy in clinical rehabilitation care in order to provide more comprehensive treatment to patients. Smart healthcare is to build a regional medical information platform for health records and use the most advanced Internet of Things technology to realize the interaction between patients and medical staff, medical institutions, and medical equipment, and gradually achieve informatization. At present, intelligent medical treatment has been widely used in the medical field, such as remote consultation, remote surgery, and AI-assisted treatment, and has successfully solved the problem of interaction between patients and multiple parties, and it achieved good results.

With the rapid development of domestic medical level today, more attention has been paid to the clinical rehabilitation of patients. COPD is a chronic bronchitis and/or emphysema with characteristics of airflow obstruction, which can further develop into lung common chronic diseases of heart disease and respiratory failure. The application of intelligent medicine to meta-analysis of clinical rehabilitation nursing of patients with COPD also has far-reaching significance for the development and expansion of clinical rehabilitation nursing of patients with COPD. The application range of intelligent medicine is very wide. In recent years, scholars have conducted research on intelligent medicine, but there are relatively few studies on the meta-analysis of intelligent medicine in clinical rehabilitation nursing of COPD patients. Therefore, this paper applied intelligent medical method to the meta-analysis research of clinical nursing of COPD patients, which had both theoretical and practical significance.

As the society pays more attention to domestic medical care, more and more scholars have done research on the meta-analysis of clinical rehabilitation nursing of COPD patients. In recent years, Fu C comprehensively analyzed the available evidence on the efficacy of HFNC on exercise capacity, lung function, and other factors related to pulmonary rehabilitation in COPD patients in the article [1]. But the data used in this analysis were not new enough. Cicotti found that the ambient intelligence (AmI) paradigm had been increasingly used to build ambient intelligent medical software (AmI-ms) to face the complexity of software-based system design [2]. But there was no strong data applied in this research to support the thesis. Before that, Zhang designed and implemented a secure medical big data ecosystem based on the Hadoop big data platform to improve the intelligence of the medical system [3]. But the system designed was not very efficient. Later, based on the intelligent medical system, Wu constructed a convolutional neural network-based auxiliary diagnosis model for staging of non-small cell lung cancer [4]. But the model designed was not put into practice. Later, Wei proposed an improved IMAD based on decision tree with low ability of intelligent auxiliary diagnosis [5]. But the theoretical foundation built in the research was not full enough. Subsequently, Ali proposed that the intelligent medical platform was a dialogue-based medical decision-making system that provided medical guidance and recommendation services based on incremental learning methods [6]. But the system did not meet the actual demand problem. By analyzing the research results of the above scholars, Jagadeesh Kumar et al. further conducted a rich intelligent medical analysis based on the facts and deep belief network learning of unlabeled vertices [7]. But there was no good conclusion being given in this analysis. Although these studies have promoted the research on clinical rehabilitation nursing of COPD patients to a certain extent, less research has been done on it.

The innovations of this paper are as follows. (1) In the clinical rehabilitation of COPD patients, intelligent medicine can be used to conduct its meta-analysis research to make the research results more comprehensive and specific. (2) By analyzing the performance of different benchmark models, it is concluded that the SCNet benchmark model is suitable for the study of this paper, and then it is analyzed for the research topic of this paper. Statistics are also used to analyze the two groups of rehabilitation nursing patients.

## 2. Meta Method of Clinical Rehabilitation Nursing of COPD Patients Applying Intelligent Medical Treatment

### 2.1. Intelligent Medical Auxiliary Diagnosis System

The concept of artificial intelligence was first proposed in 1956. After continuous development and evolution, artificial intelligence has been applied in various fields. It is a new technical science about the study of human intelligence. Among them, medical treatment is one of the fields where artificial intelligence and practice are most closely integrated. The smart healthcare assistant diacrisis system is the product after the combination of the two, which first appeared in 1972 (AAPHELP system). Its main purpose is to improve the work efficiency and clinical competence of doctors. Its core is to accomplish the processing of iatrical data and the extraction of iatrical knowledge through artificial intelligence technology. Smart healthcare mainly covers online and offline systems [8], as shown in Figure 1.

The overall structure of the interactive intelligent auxiliary diagnosis model and the detailed implementation details of each part are shown in Figure 2. The model receives the information entered by the user in the process of interacting with the system and then recommends the action in the current state. If the recommended action is a *check item*, the model will wait for the data input by the user and continue the interaction process with the user; if the recommended action is *diagnosis disease results*, the model thinks that the current interaction process can end and give the diagnosis results [9].

Among them, the smart healthcare based on iatrical images has become a hot topic, and it is the most intelligent auxiliary diagnosis system in the current practical application [10]. This is mainly because medical imaging data are the main data in medical data, and the rapid development of deep learning technologies such as convolutional neural networks has also promoted medical imaging research. The diagnosis process of intelligent medical treatment is shown in Figure 3.

This system is composed of peripheral medical equipment, intelligent medical management and service intelligent terminals, communication access network, and health service platform. The system can be used in the following aspects: reading peripheral medical equipment data information, reading patient identity information, entering doctor follow-up information, calling and viewing health files, medical management and service business operations, active push of service information, etc. [11], specifically as shown in Figure 4.

Aiming at the extraction of various modal information by the intelligent medical system, this paper used the attention mechanism to realize the key feature extraction of text features *C*_*Y*_ and obtain key text feature information *C*_*Yatt*_*ϵT*^*M*^. Because the neural attention mechanism can give a neural network the ability to focus on a subset of its inputs (or features). Its specific calculation formula is as follows:

(1) $$\begin{array}{c} R=TANH\left(EC_{Y}^{Y}+N\right), \end{array}$$

(2) $$\begin{array}{c} E_{TATT}=SOFTMAX\left(R\right), \end{array}$$

(3) $$\begin{array}{c} C_{TATT}=\overset{K}{\underset{O}{\sum }}E_{YTATT}^{O}C_{Y}^{O}, \end{array}$$

where *E* ∈ *T*^*M*^ is the training parameter, *C*_*Y*_^*Y*^ is the transpose of *C*_*Y*_, *N* is the bias, and *R* ∈ *T*^*K*^ represents the score of *K* sequence steps in the sequence *C*_*Y*_.

Then, *V*_*ATT*_ is used as the weighted feature map, in which *XC*_*IT*_ is the multimodal feature representation of the fusion image and text. The formula obtained is:

(4) $$\begin{array}{c} V_{ATT}=E_{IT}\times V, \end{array}$$

(5) $$\begin{array}{c} E_{IT}=G\left(C_{IT}\right). \end{array}$$

The feature map weight function is calculated through the fusion features *C*_*IT*_ of each modality. However, considering that different feature channels focus on different image information, this model obtains the corresponding weight of each feature channel in the image through the constructed feature channel screening network, in order to focus on the feature channel that is more relevant to the target information [12]. Its structure is shown in Figure 5.

Finally, the learned weights are normalized to obtain the final weights *E*_*IT*_, where *E*_1_ and *E*_2_ are the training parameters in the fully connected layer.

(6) $$\begin{array}{c} S=RELU\left(E_{1}\left[C_{O},C_{TATT}\right]\right), \end{array}$$

(7) $$\begin{array}{c} E_{IT}=SIGMOID\left(E_{2}S\right), \end{array}$$

Then, *C*_*G*_ ∈ *T*^2*L*^ represents the multi-modal fusion vector of 2L dimensions, and finally get:

(8) $$\begin{array}{c} C_{G}=\left[C_{1},C_{2}\right]. \end{array}$$

*YO* represents the cancer samples correctly classified by the model. *YM* represents the cancer-free samples correctly classified by the model. *GM* stands for cancer-free samples misclassified by the model [13]. *GO* represents cancerous samples misclassified by the model.

(9) $$\begin{array}{c} S_{CC}=\frac{YO+YM}{YO+TN+GO+GM}, \end{array}$$

(10) $$\begin{array}{c} G1_{SCORE}=\frac{2YO}{2YO+GO+GM}, \end{array}$$

(11) $$\begin{array}{c} Den=\frac{YO}{YO+GM}, \end{array}$$

(12) $$\begin{array}{c} D_{PE}=\frac{YM}{YM+GO}. \end{array}$$

### 2.2. Clinical Rehabilitation Nursing of COPD Patients

The main clinical symptom of COPD is chronic bronchitis with persistent airflow limitation, and even more severe patients may develop emphysema. In addition, the treatment period of COPD is long, and current moderate exercise, smoking cessation, and pulmonary rehabilitation training can improve the lung function of patients [14].

How important is rehabilitation care for COPD patients? Two sets of data were taken out for comparison. Before nursing, *P* > 0.05, after nursing, the lung function was obviously improved, *P* < 0.05. The details are shown in Table 1.

The following is a comparison of the nursing satisfaction of the two groups of patients. The nursing satisfaction of the research group was 92%, which was significantly better than that of the control group, which was 68%, *P* < 0.05, as shown in Table 2.

In addition, a cognitive questionnaire survey was conducted on patients with COPD in a hospital. The scale was orthogonally rotated by the maximum variance method to extract two common factors, namely, the cognition of self-disease management (F1) and the perception of COPD disease cognition (F2). The eigenvalues of the two common factors were greater than 1, and the cumulative contribution rate was 55.28%, indicating that the validity of the questionnaire was good, and the data collected through the questionnaire could accurately reflect the real status of the respondents' cognition of their own diseases, as shown in Tables 3 and 4.

The question setting is based on the severity of the disease, the treatment method of the disease and the current disease situation.

Most patients do not understand their own conditions and treatment, and lack understanding of their own management [15].

Pulmonary rehabilitation is an individualized comprehensive intervention after a comprehensive assessment of the patient's condition, which mainly includes exercise training, health education, psychological intervention and nutritional support. It aims to improve the physical and psychological status of patients with chronic respiratory diseases. At present, pulmonary rehabilitation is mainly used for chronic obstructive pulmonary disease [16]. Studies have confirmed that pulmonary rehabilitation training can significantly improve the exercise capacity and quality of life of patients with COPD. Below is a mind map of regular COPD patient care, as shown in Figure 6.

### 2.3. Calculation of Medical Knowledge Base

It mainly writes about the calculation method of entity and attribute distribution. If there are more web pages of two entities, the more they are related [17].

When estimating variable distribution, it is judged by the distribution of variable samples. To solve this problem, a prior distribution needs to be added. It is not related to the test results; it reflects the knowledge of other parameters *θ* before the statistical test is carried out. The resulting distribution. In the absence of any superfluous knowledge, the simplest prior distribution is the mean distribution. If the variable value is generated *L* times in advance, and then combined with the sample, this is the estimation of the distribution [18]. Therefore, the formula for calculating the prior probability of disease is Formula (13). Among them, *G*_*DI*_ is the number of diseases with serial number *O*, and the value of *L* is 10.

(13) $$\begin{array}{c} \left(O_{DI}\right)=\frac{\left(G_{DI}+L\right)}{\sum \left(G_{DI}+L\right)}. \end{array}$$

The symptom is similar to diseases, which is calculated as:

(14) $$\begin{array}{c} O\left(SI\right)=\frac{\left(G_{SI}\right)}{\sum \left(G_{SI}+L\right)}. \end{array}$$

In the case of statistical disease K, the probability of symptom O occurring is:

(15) $$\begin{array}{c} \text{O}\left(H_{O}\right)=\frac{G_{HO}}{\sum GH_{O}}. \end{array}$$

The probability of knowing the gender according to the above is the Formula (16), which *GH*_0_*F*_*K*_ means having a disease *K* and gender O. The value of *L*_3_ is 2.0.

(16) $$\begin{array}{c} \left(\left.GH_{O}\right|F_{K}\right)=\left(GH_{O}F_{K}+L_{3}/\sum \left(GH_{O}F_{K}+L_{3}\right)\right). \end{array}$$

For age, this paper divided it into 7 intervals. According to different standards, there are different ways to divide age, and the main reference here is the classification method of Google Health. For example, a newborn baby was more important for a few days and a few months. If there was enough data, the statistics of age could be made to a very precise level. But because the current data volume was not much, it could only be divided into 7 intervals [19]. They are infants, child, juvenile, young people, adult, middle-aged, and senior citizen, as shown in Table 5.

If *G*_*AI*_ represents the figure of emergence of age team *O*, there is:

(17) $$\begin{array}{c} O\left(HI\right)=\frac{G_{HI}}{\sum G_{HI}}, \end{array}$$

(18) $$\begin{array}{c} O\left(H_{I}\left|S_{K}\right.\right)=\left({GH}_{I}S_{K}+L_{4}/\sum \left(GH_{I}S_{K}+L_{4}\right)\right). \end{array}$$

After determining the respective distributions of the two parts, their results are weighted and combined. The relationship between disease and symptoms, which is the most complex relationship, is used as an example to illustrate. The following formula is obtained:

(19) $$\begin{array}{c} O\left(D_{I}\left|F_{K}\right.\right)=\frac{\alpha *O_{1}\left(\left.D_{O}\right|F_{O}\right)+\left(1-\alpha \right)*O_{2}\left(D_{O}\left|F_{K}\right.\right)}{\sum_{K}\alpha *O_{1}\left(\left.D_{O}\right|F_{O}\right)+\left(1-\alpha \right)*O_{2}\left(D_{O}\left|F_{K}\right.\right)}, \end{array}$$

where *O*_1_(*D*_*O*_|*F*_*O*_) represents the distribution obtained from structured data, and *O*_2_(*D*_*O*_|*F*_*K*_)represents the distribution obtained from the statistical data of the cases.

The final assumption is that *YG* refers to the frequency of diseased words. ofg refers to inverse document frequency. For word *Y* and document *F*, the word frequency is calculated as:

(20) $$\begin{array}{c} YG\left(Y,F\right)=0.5+0.5\times G_{T,F},/\text{MAX}\left\{G_{Y,F},F:Y\in F\right\}. \end{array}$$

## 3. Meta Experiment of Clinical Rehabilitation Nursing of Patients with Chronic Obstructive Pulmonary Disease Based on Intelligent Medical Treatment

### 3.1. Current Situation of Clinical Rehabilitation Nursing Medical Service Terminal Products for Patients with Chronic Obstructive Pulmonary Disease

At present, the research and development of domestic medical service terminal equipment is in a stage of rapid development, but the terminal equipment is generally less intelligent in patients with different diseases, and it has some defects in system interaction and function. Such as fewer self-service terminals, outdated or idle terminal functions, etc. [20].

In 2018, the number of domestic hospitals reached 30,000. Currently, some hospitals in developed eastern coastal cities use self-service terminals more, while in some third- and fourth-tier cities, the penetration rate of self-service terminal equipment is very low. As shown in Figure 7, from 2012 to 2018, the domestic medical terminal equipment holdings and the number of domestic hospital self-service terminal equipment reached 688,000 in 2018, of which the largest share and single-function automatic registration machine has reached 192,000, with a market share of 28%, while there were only 86,000 all-in-one terminals with comprehensive functions and more comprehensive services, and the market share was only 12%. It can be seen that the domestic self-service terminal equipment is still in its infancy, and most of the equipment is only satisfied with the most basic registration functions [21]. This is because the technology development and production capacity in the initial stage have not kept up.

### 3.2. Meta Experiments with Benchmark Models

In order to make a better meta-analysis of clinical rehabilitation care of COPD patients, this paper proposes a benchmark model SCNet and compares it with other models, fully demonstrating its superiority. First, in order to prove that the model proposed in this paper (SCNet) has superior performance compared with single-modal models based on text or image data, in this paper the SCNet model is experimentally compared and analyzed with the single-modal benchmark models for images and text [22]. The results are shown in Figure 8. The experimental results of each model on accuracy, specificity, sensitivity and F1-Score are shown, respectively. SCNet outperforms image classification benchmarks on Acc, Spe, Sen, as well as comprehensive metrics F1-Score and AP. This is because SCNet is stronger than other models in feature extraction. For example, SCNet is about 9% higher than the best model in accuracy. On the comprehensive index AP, compared with the curves of other models, the PRC curve of SCNet is closest to the coordinate (1, 1), and the AP value is much higher than that of each image classification benchmark model. This shows that the model designed in this paper can achieve better model performance than traditional image classification models.

In the comparison experiment between the SCNet model and the text classification benchmark model, this paper selects the CNN-based text classification model (Text_Cnn), the bidirectional LSTM model and the GRU + attention model as the comparison objects. It can be seen from Figure 9 that SCNet performs better than the text classification benchmark model on Acc, Spe, and Sen and the comprehensive indicators F1-Score and AP. For example, SCNet outperforms the best model by 2% in accuracy. On the composite metric AP, the AP value outperforms the best text classification benchmark by 3%. This shows that the model designed in this paper has a better model effect than the traditional text classification model.

In order to further prove the superiority of the SCNet model, this paper conducts an experimental comparative analysis between SCNet and the multimodal benchmark model. Figure 9 shows the experimental comparison results between the SCNet model and the GatemultimodalUnite model, the Avg_Pro model, and the Con model. It shows the experimental comparison results of each model in terms of accuracy, specificity, sensitivity and F1-Score. It also shows the PRC curve of each model and its area under the curve AP value. It can be seen that SCNet is superior to other models in all aspects, and the area under the AP value reaches 0.9374.

First, it can be seen from the figure that the accuracy of the SCNet model is better than that of the benchmark model. On the sensitivity metrics in Figure 10, SCNet outperforms the baseline model. Secondly, in the comparison of comprehensive index F1-Score and AP value, SCNet is the best performing model among all models. Although on specificity metrics SCNet does not perform the best, which is about 1% lower than the best baseline model, the comprehensive performance of the SCNet model on Acc, Sen, F1-Score, and AP indicators can show that the model SCNet proposed in this paper has certain advantages, which is helpful for the clinical rehabilitation care of patients with COPD. It also can better assist doctors to carry out treatment.

### 3.3. Meta-analysis of Clinical Rehabilitation Nursing in Patients with Chronic Obstructive Pulmonary Disease Using Statistics

In order to conduct a statistical meta-analysis of various aspects of clinical ConocoPhillips care for patients with COPD, we compared the patients as two groups.

Pulmonary rehabilitation treatment group: this group had completed various scales and scores upon admission, and they were tested pulmonary function and given basic treatment according to the guidelines. Conventional drug treatment included respiratory support, oxygen inhalation, anti-infection, expectorant, anti-inflammatory, antispasmodic, and antiasthmatic. From the second day of admission, pulmonary rehabilitation treatment, health education, sputum excretion guidance, etc. were carried out according to the pulmonary rehabilitation treatment plan until discharge. The pulmonary rehabilitation treatment was completed under the guidance and supervision of medical staff. Upon discharge, various scales and scores were completed again to test lung function [23].

Routine treatment group: This group has completed various scales and scores, and they were tested lung function and given basic treatment according to the guidelines on admission. Patients in this group could not undergo any form of pulmonary rehabilitation training during hospitalization. Upon discharge, various scales and scores were completed again to test lung function [24].

Pulmonary rehabilitation regimens were as follows. From the second day of hospitalization, Zheng's recumbent position rehabilitation exercises were performed under the direct supervision of medical staff. Before the training, full-time medical staff distributed pictures and video materials to the patients. The lying position rehabilitation exercises consisted of four movements: stretching. Sit-ups, bridge exercises, air pedaling, and abdominal pursed lip breathing.

Patients without carbon dioxide retention and those with percutaneous fingertip oxygen saturation<92% could be kept under nasal cannula oxygen inhalation, while those with carbon dioxide retention could be kept under non-invasive ventilator-assisted ventilation.

They were instructed to perform cough, expectoration, and expectoration training. It was advisable to sit or stand upright, with the upper body leaning forward slightly, while slowly pursing the lips and exhaling. After taking a deep inhalation, they should return to the upper body, contract the abdominal muscles, and use abdominal strength to actively cough. They also should cough out the air in the lungs, and stop coughing after 3–5 times in a row. If there was secretion, it should be discharged through the mouth in time and handled properly. Then the pursed-lip breathing method was used to breathe calmly for several times, or they could rest for a while. Next, the above steps were repeated. Small auxiliary instruments also can be used, such as respiratory expectoration valves, to guide effective coughing and promote the discharge of respiratory secretions.

Precautions during exercise: transcutaneous oxygen saturation and heart rate should be monitored in real time, and pulmonary rehabilitation training should be stopped immediately. The following situations should be dealt with: first, the heart rate is greater than the target heart rate (target heart rate = (220 − age − resting heart rate) × 50% + resting heart rate). If the patient did not relieve after rest or the patient's heart rate could not fall to the normal range, it was necessary to stop exercising and find the cause of the increased heart rate of the patient. The second was refractory hypoxia, which was still lower than 88% after high-flow oxygen inhalation. Third, the patient had obvious increased shortness of breath, increased dyspnea, chest tightness, chest pain, palpitations, severe headache, abdominal pain, nausea, and vomiting, or they complained of intolerance. Fourth, if the patient's blood pressure dropped significantly below 90/40 mmHg, or the blood pressure rose significantly, exceeding 180/110 mmHg, it is necessary to suspend exercise and be observed. Fifth, the patient fainted and lost consciousness.

1. Health education is also an essential part of pulmonary rehabilitation. Patient health education is usually carried out by a pulmonary rehabilitation specialist team. The main content is to educate and guide patients and their family members to urge and encourage patients to adhere to pulmonary rehabilitation exercises, and regularly follow up on their health and well-being. The implementation of the exercise program should also be supervised. Patients should be helped to change their unhealthy lifestyles and establish healthy behaviors to promote behavioral changes. At the same time, the patient's family members should be educated about the disease so that they can correctly understand the disease, treat the disease, and maintain a healthy mood. Specifically, it can be divided into the following aspects:

Firstly, disease education: the knowledge of chronic obstructive pulmonary disease related diseases needs to be explained in order to make the subjects understand the concept of disease and understand their own condition. The patients also should be guided to know the basic drugs and common side effects related to chronic obstructive pulmonary disease, especially the correct use and precautions of inhaled preparations that require long-term use. Knowledge of home oxygen therapy and mechanical ventilation, knowledge about pulmonary rehabilitation can be educated through audio-visual materials, bedside demonstrations, real-life demonstrations, etc., especially the explanation and guidance of exercise therapy, also needs to be popularized. In addition, compliance and satisfaction of patients should be satisfied and they need to be instructed to pay attention to weather changes and changing clothes in a timely manner, avoiding getting cold and preventing colds. It is also important for these patients to avoid going to crowded places to prevent respiratory infections. Moreover, they need to understand the indications for hospitalization for acute exacerbations.

Secondly, life education: the subjects should be persuaded to quit smoking and drinking, and avoid second-hand smoke to get rid of irritating gas or polluted gas environment. The connection among smoking, drinking and COPD should also be explained to them so as to help patients develop good living habits. The first point is to stay away from tobacco. Smoking can cause a variety of diseases and accelerate our aging. It can be said that there are no harms and no benefits, so smoking cessation is necessary. It not only to ensure that the patients themselves do not smoke, but also to persuade the people around them to quit smoking, jointly creating a smoke-free and harmless environment. The second point is to avoid contact with the polluted environment. If the occupation requires protection, the inhalation of harmful substances and allergens should be minimized. When cooking at home, it is necessary to try to choose healthy and nutritious methods such as cooking, and avoid deep-frying, barbecue and other methods. They need to reduce travel in hazy days and use air purifiers indoors. They must wear effective filtering masks when going out.

Thirdly, diet guide: chronic obstructive pulmonary disease patients are in a state of chronic consumption for a long time, coupled with the decline of digestion and absorption function, long-term insufficient energy intake, abnormal metabolism and so on, resulting in different degrees of malnutrition. In patients with acute exacerbation of COPD will increase consumption due to infection and stress on the one hand, and they may be led to severe negative nitrogen balance because of insufficient nutrient intake and absorption disorder due to impaired gastrointestinal function on the other hand. Therefore, reasonable nutritional support can improve lung function in patients with acute exacerbation of COPD, delay disease progression, and improve prognosis. The prevalence of malnutrition in COPD patients ranges from 20% to 60%. Malnutrition and cachexia may increase the risk of death in patients with chronic obstructive pulmonary disease. Therefore, reasonable dietary advice is of great significance.

Fourthly, psychological counseling: Others needs to establish a good relationship with patients. It is necessary to timely understand and master the patients' adverse emotional changes. Timely communication with them is significant in order to effectively ease their moods, avoiding further development of depression. These patients also should be provided with positively social and psychological support in order to help them build confidence in overcoming the disease and correctly understand diseases. In addition, to eliminate anxiety and tension in the face of illness, yoga, meditation and other training to regulate emotions can be carried out appropriately, so as to ensure high-quality and effective sleep. Therefore, a harmonious state of physical and mental balance can be achieved, improving treatment compliance and speeding up the progress of pulmonary rehabilitation.

Then all the data were analyzed by SPSS22.0 statistical software, and the data in each group was tested for normality, which were expressed as mean ± standard deviation (mean ± SD). The rank sum test was used to compare the differences between the two groups. The difference was statistically significant with *p* < 0.05. The normal distribution test showed that the difference between the experimental group and the control group did not meet the normal distribution, the statistical analysis method was paired rank sum test, and the comparison of the therapeutic effect between the laboratorial team and the control team was performed by two independent samples rank sum test.

Finally, it was found that the pulmonary function indexes of the pulmonary rehabilitation treatment group and the conventional treatment group were improved after treatment compared with those before treatment, and the differences in the degree of improvement before and after treatment were further analyzed. Among them, FEV1/FVC was the most commonly used parameter to judge whether there was expiratory airflow obstruction. There was no disparate in the degree of change in this value between the pulmonary rehabilitation treatment group and the conventional treatment group, indicating that pulmonary rehabilitation treatment could not significantly improve airflow degree of blocking in COPD patients in the short term. However, FEV1 had the best repeatability in the pulmonary function test and was also the most commonly used parameter for judging the degree of damage. The change of this index in the pulmonary rehabilitation treatment group was more obvious than that in the conventional treatment team, and the disparity was statistically valid, suggesting that short-term pulmonary rehabilitation treatment had a certain effect on delaying the damage of lung function.

## 4. Discussion

This article is devoted to the study and design of a meta-analysis of clinical rehabilitation care for COPD patients based on intelligent medicine, and applies it to the analysis of clinical rehabilitation nursing of patients with COPD. This not only expands the scope of intelligent medical applications, but it is also a new attempt to research the complexity of clinical rehabilitation and nursing care for patients with COPD. By comparing the performance of multiple models, it is determined that the model used in this paper is the most suitable for this study. It also shows that intelligent medicine is also a vital tool to study the complexity of the system and has certain potential in the study of the complexity of clinical rehabilitation nursing of patients with COPD. In addition, based on the current situation of the existing medical equipment, the analysis is carried out and the model comparison is added. Finally, the clinical rehabilitation nursing of patients with COPD is analyzed by statistical calculation. For the research of intelligent medical treatment, this paper starts with the introduction of the most basic intelligent medical system and analyzes the structure of intelligent medical treatment. At last, intelligent medicine is successfully applied in the meta-analysis of rehabilitation nursing of COPD patients. This paper uses the benchmark model to find that the best model suitable for this study is SCNet, analyzes the performance of the model in all aspects, and then compares the rehabilitation conditions of the two groups of patients.

It is shown that clinical rehabilitation care for COPD patients based on intelligent medical treatment is more effective than single rehabilitation care, and patients can interact better with medical equipment and doctors. This can greatly reduce the patient's unknown to the disease. In specific practical decision-making, hospitals can formulate different clinical rehabilitation care plans through intelligent medical care for patients with different symptoms, which makes rehabilitation treatment more effective and facilitates patients to know their own news.

This paper takes the current situation of intelligent medical equipment in a hospital as a case study. First, through statistical and qualitative analysis to determine the current state of medical equipment and comparison of the SCNet model with other groups of models, it can be known that it is the most suitable model for this study. After analysis, it is concluded that the clinical rehabilitation nursing of COPD patients based on intelligent medical treatment is very effective in terms of the degree of recovery of the patients.

## 5. Conclusions

Through the case study, important conclusions can be drawn: based on the blessing of the intelligent medical system, the clinical rehabilitation nursing of COPD patients will be more comprehensive and effective. The pulmonary function indicators of the pulmonary rehabilitation treatment group and the conventional treatment group are also better than those before treatment. But this is not absolute. For example, in the research on the current situation of medical equipment in this case, there are still many places where intelligent medical care has not been applied. This requires closer study of intelligent medical care in the future in order to conclude solution. The article is a meta-analysis research on clinical rehabilitation nursing of COPD patients based on intelligent medical treatment. The selection of this project is relatively limited, but in reality there are often more choices. In addition, the research application in reality should also be analyzed in combination with a variety of factors, which will have greater value and certainly greater difficulty. But it is undeniable that we always believe that there will be more and more research on intelligent medicine in the medical field, and the domestic medical level will also be higher and higher. The analysis of clinical rehabilitation care of patients with COPD will get better and better.

## Figures and Tables

**Figure 1:** Smart healthcare service model.

**Figure 2:** Active interactive intelligent diagnosis model framework diagram.

**Figure 3:** Diagnostic system flowchart.

**Figure 4:** System composition.

**Figure 5:** Weight generation module.

**Figure 6:** Mind map of nursing care of patients with COPD stabilizer.

**Figure 7:** Status of medical service equipment.

**Figure 8:** Comparative analysis of SCNet and image classification models.

**Figure 9:** Comparative analysis of SCNet and text classification models.

**Figure 10:** Comparison of SCNet and multimodal benchmark model experiments.

**Table 1:** Comparison of various indicators before and after nursing in the two groups.

Indicators	Observation group (*N* = 15)		The control group (*N* = 15)	
	Care before	After the nursing	Care before	After the nursing
FEV (L)	1.52 ± 0.35	1.59 ± 0.69	1.63 ± 0.38	1.49 ± 0036
FEV (%)	56.95 ± 10.29	65.42 ± 9.75	58.73 ± 10.98	62.28 ± 12.34
FVC (L)	2.04 ± 0.33	2.49 ± 0.39	2.21 ± 0.27	2.26 ± 0.31
FVC (%)	50.79 ± 11.41	66.49 ± 12.94	50.97 ± 10.98	55.49 ± 12.45
FEV/EVC	63.49 ± 11.39	74.28 ± 11.02	2.21 ± 0.27	64.25 ± 13.45
6MWT (M)	313.05 ± 41.01	423.78 ± 57.73	312.98 ± 37.55	38.19 ± 54.32

**Table 2:** Comparison of nursing satisfaction between the two groups.

Group	The number of cases	Satisfied with the number of cases	Basic satisfaction cases	Number of dissatisfied cases	Nursing satisfaction
The team	25	17	6	2	23 (92.00)
The control group	25	11	6	8	17 (68.00)
*χ* ^2^ value					4.500
*P* values					0.033

**Table 3:** Factor analysis of cognitive questionnaire for COPD patients.

Entry	F1 _	F2 _
Whether you know the severity of your own disease (COPD)	0.800 _	0.753 _
Are you aware of the medical indications for “your illness (acute exacerbation)	0.609	0.732
Do you know the treatment for your disease	0.647	0.745
Whether chronic obstructive pulmonary disease (COPD) needs long-term regular treatment	0.800	
Have lung function tests been performed		0.551
Whether annual lung function tests are required	0.531	
Do you make regular visits to the doctor		0.477

**Table 4:** Factor analysis of COPD cognitive questionnaire - overall explained variance.

Factor	The eigenvalue	Variance interpretation rate	Cumulative contribution rate
1	4.277	42.772	42.772
2	1.251	12.508	55.280
3	0.948	0.477	64.757
4	0.847	8.474	73.231
5	0.751	7.509	80.739
6	0.620	6.203	86.942
7	0.500	5.003	91.945
8	0.395	3.954	99.899
9	0.316	3.161	99.060
10	0.094	0.940	100.000

**Table 5:** Age range division.

Serial number	Age range	Designation
0	0–2 _	Infant
1	3–5 _	Child
2	6–13 _	Juvenile
3	14–18	Young people
4	19–40	Adult
5	41–60	Middle-aged
6	60+ _ _	Senior citizen

## Data Availability

No data were used to support this study.
